The article "Kidney Tumor Detection and Classification Based on Deep Learning Approaches: A New Dataset in CT Scans" was published in 2022. Journal: J Healthc Eng.

# Kidney Tumor Detection and Classification Based on Deep Learning Approaches: A New Dataset in CT Scans

**DOI:** 10.1155/2022/3861161

**Published:** 2022-10-22

**Authors:** Dalia Alzu'bi, Malak Abdullah, Ismail Hmeidi, Rami AlAzab, Maha Gharaibeh, Mwaffaq El-Heis, Khaled H. Almotairi, Agostino Forestiero, Ahmad MohdAziz Hussein, Laith Abualigah

**Affiliations:** ^1^Department of Computer Information Systems, Jordan University of Science and Technology, Irbid 2210, Jordan; ^2^Department of General Surgery and Urology, University of Science and Technology, Irbid 22110, Jordan; ^3^Department of Diagnostic and Interventional Radiology, Faculty of Medicine, Jordan University of Science and Technology, Irbid 2210, Jordan; ^4^Computer Engineering Department, Computer and Information Systems College, Umm Al-Qura University, Makkah 21955, Saudi Arabia; ^5^Institute for High Performance Computing and Networking, CNR, Rende (CS), Italy; ^6^Deanship of E-Learning and Distance Education, Umm Al-Qura University, Makkah 21955, Saudi Arabia; ^7^Hourani Center for Applied Scientific Research, Al-Ahliyya Amman University, Amman 19328, Jordan; ^8^Faculty of Information Technology, Middle East University, Amman 11831, Jordan; ^9^School of Computer Sciences, Universiti Sains Malaysia, Pulau Pinang 11800, Malaysia

## Abstract

Kidney tumor (KT) is one of the diseases that have affected our society and is the seventh most common tumor in both men and women worldwide. The early detection of KT has significant benefits in reducing death rates, producing preventive measures that reduce effects, and overcoming the tumor. Compared to the tedious and time-consuming traditional diagnosis, automatic detection algorithms of deep learning (DL) can save diagnosis time, improve test accuracy, reduce costs, and reduce the radiologist's workload. In this paper, we present detection models for diagnosing the presence of KTs in computed tomography (CT) scans. Toward detecting and classifying KT, we proposed 2D-CNN models; three models are concerning KT detection such as a 2D convolutional neural network with six layers (CNN-6), a ResNet50 with 50 layers, and a VGG16 with 16 layers. The last model is for KT classification as a 2D convolutional neural network with four layers (CNN-4). In addition, a novel dataset from the King Abdullah University Hospital (KAUH) has been collected that consists of 8,400 images of 120 adult patients who have performed CT scans for suspected kidney masses. The dataset was divided into 80% for the training set and 20% for the testing set. The accuracy results for the detection models of 2D CNN-6 and ResNet50 reached 97%, 96%, and 60%, respectively. At the same time, the accuracy results for the classification model of the 2D CNN-4 reached 92%. Our novel models achieved promising results; they enhance the diagnosis of patient conditions with high accuracy, reducing radiologist's workload and providing them with a tool that can automatically assess the condition of the kidneys, reducing the risk of misdiagnosis. Furthermore, increasing the quality of healthcare service and early detection can change the disease's track and preserve the patient's life.

## 1. Introduction

The kidneys in the human body cleanse waste products and pollutants from the blood [1, 2]. The abnormal growth of cells causes tumors (cancers), affects people differently, and causes different symptoms.

Therefore, the early detection of kidney tumors (KT) is an essential step to reduce the risk of further disease progression. Consequently, this leads to the patient's life preservation [2, 3]. Although around a third of KT cases are discovered after being spread to other areas, most conditions do not induce symptoms. They are often found when the patients are being treated for other diseases. Kidney tumors can be observed accidentally on radiography and may appear as masses, kidney cysts, or abdominal pain in patients. The signs likely have nothing to do with the kidneys [4, 5]. However, low hemoglobin, weakness, vomiting, stomach pain, blood pee, or high blood sugar are among the most subtle symptoms or infections KT causes. Also, anemia occurs in about 30 percent of patients with KT [6, 7]. Unfortunately, tumors and solid masses that can arise inside the kidneys are often cancerous. The value of determining the presence of the tumor is to choose the appropriate method for treatment; hence, the rate of recovery from the disease may depend on the early detection of the tumor. One of the necessary tests to determine the tumor is computed tomography (CT) scans of the abdomen and pelvis to the patients, which have characteristics studied to judge whether the kidney has a tumor.  Figure 1 shows a case of KT, a renal mass lesion in the left kidney measuring about 4 cm besides 3D volume rendering of the kidneys (kidney in pink and renal cancer in blue). A tumor threatens a person's life, so many procedures resolve this obstacle through accurate tumor diagnosis [8, 9].

Deep learning (DL) is one of the most powerful machine learning technologies that can automatically learn multiple features and patterns without human intervention [10–12]. DL enabled the building of predictive models for the early diagnosis of tumor disease, and scientists used proven pattern analysis methods. DL algorithms outperformed traditional machine learning due to their highly accurate results [13–15]. Also, it often matches or surpasses human performance. That is why they are recommended as the best method for dealing with images [16, 17]. It has gained attention in image processing, especially in the medical field, because radiology is primarily concerned with extracting useful information from images.

Object detection is the method of identifying the class instance to which the object belongs. There are several types of detection, such as single-class object detection and multiclass object detection [18]. Object detection has been applied in a wide field of medical images because of its precise effect on discovering diseases of all kinds. The convolutional neural network (CNN) is widely used to extract image characteristics and detect different objects. It is a neural network that operates on the principle of weight sharing. The convolution is an integral part of a function that explains how one function interferes with another. The size and the number of images, the number of working layers, and the form of activation functions used in CNNs vary [19]. Variables of CNNs are selected experimentally and on a trial-and-error basis. Besides, every CNN consists of several layers, the most important of which are the convolutional and subsampling (pooling) layers [20].  Figure 2 shows an illustration of CNN architecture.

Over the years, many variants of CNN structures were developed to solve difficult real-world problems and obtain sufficient accuracy. In our study, we have applied VGG16 and ResNet50, besides two modified CNNs. Qassim et al. developed a CNN-based network model, VGG16, that achieved 92.7% top-5 test accuracy in ImageNet. ImageNet-2014 is a competition with approximately 15 million high-resolution images that have been classified into roughly 22,000 categories. The VGG16 network consists of 16 layers that have weights, 13 convolutions (cov) and 3 fully connected (FC) layers besides its learning time of 16.55 ms. The image entered into the cov1 layer has a fixed size, which is 224 × 224. The image is scrolled through a set of layers, where filters 3 × 3 were used and also 1 × 1 convolution filters. The convolution step is fixed at 1 pixel so that accuracy is maintained after torsion. Max-pooling is performed via a 2 × 2-pixel window. Also, three fully connected (FC) layers follow a stack of convolutional layers. The final layer is the softmax layer. The composition of fully connected layers is the same in all networks. All hidden layers are equipped with a calendar ReLU [21].  Figure 3 shows the architecture of the VGG16 model. In addition, the ResNet50s is an improved version of convolutional neural network developed in 2015. This network consists of 50 layers, 49 convolutions and one fully connected layer. Each convolution block has three convolution layers besides its learning rate of 12.83 ms. The image entered into the cov1 layer has a fixed size, which is 224 × 224 [22].  Figure 4 shows the architecture of the ResNet50 model.

Moreover, this paper has collected a novel dataset, renal CT scans, consisting of 8,400 frames. As a preliminary study on the new dataset, a convolutional neural network (CNN) framework with six layers has been proposed to diagnose tumors. Then, a CNN framework with four layers has been proposed for classifying the tumor type. We have confined CNN's training process and directed the CNNs to generate anatomically more viable predictions, mainly when the input picture data are not clear enough (e.g., missing object edges and boundaries). In addition to our proposed model's architecture, we have used state-of-the-art networks in the study, which are the ResNet50 with 50 layers and VGG16 with 16 layers [21]. Finally, we evaluate and test our model on the new renal CT for 2020 and 2021.

The remainder of this paper is organized as follows.  Section 2 presents the related work to detecting CT images.  Section 3 describes the materials, including data set collection and description.  Section 4 describes the methods, including data preprocessing, augmentation, and network architectures. Also, Section 5 shows the experiments and results. Lastly, Section 6 presents the discussion and conclusions.

## 2. Related Studies

This section begins with a discussion of works of literature, each of which addresses the issue of early KT detection and classification using various machine learning and deep learning techniques based on CT scans.

Ghalib et al. [23] conducted a study for renal tumor detection using deep learning approaches on CT scans. The authors developed an efficient algorithm to detect and further analyze renal cancer tumors using CT for patients. The preprocessing technique involved identifying the noises of a CT scan and removing them with a proper filtering technique. Image enhancement is also performed using contrast-limited adaptive histogram. The classification process is determined based on the patterns of visual appearance that include contrast, size, location, surface area, color, volume, risk, specialization, density, and risk. Based on their experimental results, the proposed model obtained high performance in classifying tumors into normal and abnormal, achieving 0.85 sec of average execution time.

On the other hand, Liu et al. [24] conducted a study for exophytic renal tumor detection through machine learning techniques on CT scans. They used 167 CT scans and developed a framework for kidney segmentation on non-contract CT images using efficient belief propagation. Based on their experimental results, the proposed model obtained high performance with 95% and 80% rates of sensitivity of exophytic lesion and endophytic lesion detection, respectively.

Furthermore, Mredhula and Dorairangaswamy [25] conducted a study for KT detection and classification using deep learning approaches and traditional machine learning techniques on CT scans. They used 28 CT scans for different categories of kidney tumors, where the used dataset was acquired from their database. They focused on implementing a semiautomatic segmentation method, defining that the segmentation of the gray-level images provides information such as the anatomical structure and the identification of the region of interest to locate tumors. Besides, they proposed an associative neural network (ASNN) model that combined the *k*-nearest neighbor (KNN) technique with an ensemble feedforward neural network.

Lately, Zhou et al. conducted a study about differentiating renal tumors based on deep learning [26]. To investigate the effect of transfer learning on CT, they used 192 CT scans for patients to differentiate between benign and malignant tumors and attempted to improve the accuracy by building patient-level models. The CNN architecture used was cross-trained InceptionV3 to perform the classification task. Five image-level models were established for each of the slices. The performance evaluation of the model was performed using the receiver operating characteristic metric on five-fold cross-validation. The results showed high accuracy with a 97% rate. The researchers concluded that deep learning approaches are useful for renal tumor classification based on CT scans and recommended benefiting from 3D CT scans to achieve more accurate results.

More recently, Zabihollahy et al. [27] conducted a study about the detection of solid renal masses using deep learning approaches on CT scans. They used semiautomated majority voting 2D-CNN, fully automated 2D-CNN, and 3D-CNN to classify RCC from benign solid renal masses on contrast-enhanced computed tomography (CECT) images. They used CT scans for 315 patients, in which the dataset included 77 scans for patients with benign solid renal masses and 238 scans for patients with malignant renal masses. They generated slices of scans manually and utilized the CNN model to extract features from each slice. Then, the classification was performed using the aggregation of CNN predictions and evaluated by the majority voting technique. Based on their experimental results, the proposed model obtained high performance with 83.75%, 89.05%, and 91.73% rates of accuracy, precision, and recall for the classification between RCC and benign tumors, respectively.

Also, Schieda et al. [28] conducted a study about the classification of solid renal masses using machine learning techniques on CT scans. They have used CT scans for 177 patients with solid renal. The features were extracted through manual segmentation with radiologists from three phases of scans: nephrographic phase contrast-enhanced, corticomedullary, and non-contrast-enhanced. The proposed method utilized the XGBoost machine learning technique. It was used to generate classifiers and, simultaneously, to search for the collection(s) of texture features that accurately discriminated between outcomes. The proposed model obtained high performance with 0.70 rates of AUC in classifying renal cell carcinoma from benign tumors and 0.77 rates of AUC in classifying clear cells of RCC from the other types.

Finally, Yap et al. [29] conducted a study about the classification of renal masses using machine learning technique CT scans. They used CT scans for 735 patients with renal masses, in which the dataset included 196 scans of benign masses and 539 scans of malignant cases. They segmented scans manually by utilizing the 3D Synapse 3D tool by cooperating with two expert radiologists, where the features were extracted based on shape and texture matrices. The proposed methods used two machine learning techniques, which are AdaBoost and Random Forest. Based on their experimental results, Random forest obtained high performance on both features with 0.68 to 0.75 rates of AUC for the classification of renal masses.

## 3. Dataset

This section focuses on the data collection process and data analysis.

### 3.1. Data Acquisition and Preparation

This work presents new data consisting of images and text “ metadata” obtained from KAUH hospital in Jordan. In this paper, we worked on the image data. The current study has collected scan data for renal masses cases from the hospital's database, performed by the interventions computed tomography (CT) scan service. Although the image set provides more than one picture from different dimensions for each patient, the diversity of images helps us get an accurate diagnosis. Besides, clinical text data support our findings and help us understand the collected images. From these miscellaneous data, different studies can be conducted. The collected dataset consists of 8400 images of 120 adult patients who have performed a CT scan for suspected kidney masses. The images are provided in (DICOM) format, considered the most standard for the interchange and transmission of medical images used worldwide. The data collected included a CT scan with contrast material and without contrast.  Figure 5 shows a sample CT with contrast and without contrast taken from the dataset.

For comparing the current dataset with the available public dataset, Table 1 summarizes the public datasets of renal CT scans for diagnosing kidney tumors by showing their sizes and sources. For example, the G037-RCP dataset exported by the Royal College of Pathologists (RCPath) located in London combines multihealth data, such as texture, images, tests, and educational information. The C4K-KiTs19 dataset is an abbreviation for Climb 4 Kidney Cancer collected from the University of Minnesota Medical Centre [31]. The TCGA dataset is an abbreviation for the Cancer Genome Atlas, which is a cancer program that has data samples spanning 33 cancer types [37]. Besides, the CPTAC-CCRCC program investigated 110 tumors regarding the TCIA dataset. The current study's dataset exceeds the other datasets regarding size, number of patients, and diversity of images. It is considered the first collected data from Jordan's King Abdullah University Hospital (KAUH). The CT scan images and metadata were collected manually and supervised by a specialist team. There are 70 CT scans for each patient. It is strongly believed that this dataset can be the basis for subsequent studies to diagnose tumors and stones, cysts, and any kidney problems, such as inflation, infection, and hydronephrosis. The proposed dataset will be publicly available for researchers up to their request (https://github.com/DaliaAlzubi/KidneyTumor).

### 3.2. Data Set Annotation and Visualization

Data were collected for adult patients between the ages of 30 *±* 80, 55 females, and 65 males, who underwent CT images of the abdomen and pelvis. Of 120 patients, 60 tumors were classified as benign or malignant and 60 cases were diagnosed as normal cases without tumors. Still, half of the normal cases suffer from cysts, hydronephrosis, and stones. Also, some of them suffer from cancers in neighboring organs such as the colon, liver, breast, lung, stomach, and their condition for follow-up.

Therefore, they must perform a CT scan periodically to ensure that cancer in other organs has not spread to the kidneys. Besides, some cases are suffering from a nephrectomy or part of it due to RCC, and their condition must be monitored to ensure the safety of kidney function and that the tumor does not spread.  Table 2 and Figure 6 show an analysis of the gender situation for all cases in the dataset.

The clinical observations include ID, age, gender, date of the scan, patient history, symptoms, diagnosis, type of right kidney injury, type of left kidney injury, both kidney disease segmentation, tumor stage, patients situation if they have a tumor or it is a normal case completely healthy or normal case with a cyst or stone. Also, they include the tumor type: Benign or Malignant, the Subtypes of the tumor, and the Test.

All patients had a CT multidimensionally examined for the pelvic and abdominal area that outlined various slices of the renal, ureter, and bladder region. These metadata were constructed and labeled manually based on the clinical reports. The data were reviewed by radiologists and the medical staff of the kidneys and urinary tract. In cooperation with them, the correctness of the data structure was checked and validated. The dataset contains (20) attributes and numerical and categorical data that describe all dataset characteristics, as shown in Table 3. In addition, the patient's data are divided into categories.

The “Situation” attribute illustrates the patient condition as three labels: Normal case “healthy” (1), Normal case with cyst (2), and Tumor (3), as shown in Table 4.

The “Tumor Type” attribute illustrates the tumor type as two labels: Malignant (1) and Benign (2), as shown in Table 5.

The “Taking Contrast” attribute illustrates if the patient has taken Contrast material as two labels: Yes (1) and No (2), as shown in Table 6.

The “Tumor Class” attribute illustrates the tumor class as five labels: Adenoma (1), Angiomyolipomas (2), Lipomas (3), RCC (4), and Secondary (5), as shown in Table 7.

The “Stage” attribute illustrates the grade of the tumor as four labels: I (1), II (2), III (3), and IV (4), as shown in Table 8.

The “Segmentation Injury in Right Kidney” and “Segmentation Injury in Left Kidney” attributes illustrate the location of the tumor: upper, middle, lower, healthy, and undefined, as shown in Table 9.

Regarding the statistical analysis of the collected data for kidney patients, 83 cases were taken in 2020 and 37 cases were taken in 2021.  Figure 7 shows the age of normal and tumor cases; for normal cases, there are 3 cases for patients between 30 and 40 years old. For 40–50 years old, there are 9 cases, 25 cases for 50–60 years old, 12 cases for 60–70 years old, and for 70+ years old, there are 11 cases. And for tumor cases, between 30 and 40, there are 5 cases; between 40 and 50, there are 6 cases; between 50 and 60, there are 19 cases; between 60 and 70, there are 14 cases, and 70+ there are 16 cases.

Contrast material is given to the person to be examined by X-ray imaging to enhance the quality of the image. Thus, that is easy for the doctor to distinguish between healthy injured tissues, facilitate the distinction of blood vessels, and determine the extent of their injury [38].  Figure 8 shows the patients who had taken contrast material before the CT test for normal cases, where 35 had taken contrast and 25 had not. And for tumor cases, 38 had taken contrast and 22 had not. Based on the above analysis, a patient who was not given a contrast had allergies, diabetes, impaired kidney function, and kidney dialysis. In addition, it is considered a risk factor because of its harmful effects such as nausea, vomiting, high or low blood pressure, caused itching, sensitivity or shortness of breath, or problems with breathing or heart failure.

Figures 9 and 10 show the classification of tumor type and subtype for all tumor cases. Of the 60 tumors cases 38 are divided into benign and 22 malignant. For benign cases, there are 28 cases considered adenoma that can be excised and treated; nine angiomyolipoma cases must be removed because they are considered a hemorrhagic cyst, and one case is considered lipomas. Besides, for malignant cases, 11 are considered RCC and 11 cases are considered metastasis due to the transfer of the tumor from neighboring organs. In adenomas cases, most of them suffered from pressure, diabetes, and liver problems such as cysts and tumors. Also, secondary cases suffered from cancers in other organs such as breast, colon, and right kidney nephrectomy because of RCC, ureter, and uterus.

The incidence of different tumor types is linked to gender differences, and it is also related to the treatment method because it does not have the same response.  Figure 11 shows the gender and the tumor classification. It is clear that most cases of kidney tumors are in men. The percentage of males having tumors is higher than that of females. In addition, males reach a later stage of the tumor than females because the rate of smoking in men is higher than that of women. Also, the tumor spreads in men more quickly than it spreads in females.

According to the statistical analysis of the gender affected by the tumor that is shown in Figure 11, the results prove the truth of the information in the National Cancer Institute (NCI) since men are more likely than women to develop tumors. The institute reports that one out of every two men and one out of every woman will develop cancer during their lifetime [39].

Figure 12 shows a statistical analysis of the location of the tumor. For the left kidney, there are 21 cases in the upper, 17 cases are healthy, 11 cases in the lower, and 9 cases in the middle. While on the other hand, for the right kidney, there are 24 cases of healthy, 18 cases in the upper, 8 cases undefined, 7 cases in the lower, and one case in the middle. Based on these analyzes, we found that most of the tumors in the right kidney are located in the upper part, and the lower part and most of the tumors in the left kidney are located in the upper, middle, and lower parts. The healthy label means that there is no tumor in this kidney. It is possible that the tumor is in one kidney and the other is healthy. The undefined label means that this kidney may have been partially or completely nephrectomy, or it may be that the expert is unable to diagnose the location of the tumor, or it may be that the scan is not clear enough to determine the exact location of the tumor due to not taking the contrast material or because the patient moved during the CT test.

Figure 13 shows the tumor stage for all tumor patients, where there are 55 cases in the first stage, two cases in the second stage, two cases in the third stage, and one case in the fourth stage. Thus, most tumors are in the I stage, meaning that they can be treated, and there are some cases in the late stage, which is a threat to the patient.

## 4. Methodology

This section describes our proposed methodology for KT detection and classification using CT scans. It includes a detailed explanation of our preprocessing steps and the used data augmentation techniques and an illustration of the architecture of the four models we built for KT diagnosis. We examine the patient's situation and define tumor presence to reduce the harmful effects of the injury and reduce the number of deaths and define the tumor type. Therefore, we have collected the new dataset from (KAUH) that contains images and metadata. We have also used the OpenRefine tool and tableau for preprocessing step to have a cleaned dataset. Furthermore, we used a DICOM converter to change the image format, and we have chosen 70 images of the kidneys from different dimensions for each patient.  Figure 14 shows the workflow of the proposed framework.

We built prediction networks, three models to make multidiagnosis for the classification of different 4 labels revolving around two phases. In the first phase, we classify the case as normal case or tumor case, while in the second phase, we classify the tumor detected as benign tumor or malignant tumor where artificial neural network modeling is used where neurons correspond to receptive fields similar to neurons in the visual cortex of a human brain. These networks are very effective for tasks of detection, categorization of objects, image classification, and segmentation. The goal of CNNs is to learn higher-order characteristics using the convolution operation. Since convolutional neural networks learn input-output relationships (where the input is an image), the output is a feature map (image class label).

In this study, we examine the patient's situation and define tumor presence to reduce the harmful effects of the injury and reduce the number of deaths. Therefore, we have collected a new dataset from (KAUH) that contains images and metadata. We have also used the OpenRefine tool and tableau to make some preprocesses steps to have a cleaned dataset. Furthermore, we used a DICOM converter to change the image form, and we have chosen 70 images of the kidneys from different dimensions for each patient. Then, we started by implementing a convolutional neural network for binary classification with the labels (Normal/Tumor).

Artificial neural network modeling is very effective for detecting tasks, categorization of objects, image classification, and segmentation. The goal of CNNs is to learn higher-order characteristics using the convolution operation. Since CNN's learns input-output relationships (where the input is an image), in convolution, each output pixel is a linear combination of the input pixels [40].

We aim to implement a binary classification solution for the detection of kidney tumors. The use of CNN in such a case helps to identify the feature map for each image engaged in the tanning process for the adopted CNN model. Hence, the use of the pooling layer helps to determine the size of the feature segment that we are looking for to extract a featured image, which will be the primary feed data into the fully connected neural network in the CNN model. As represented in Figure 15, we have two classes to be trained on it.

The study aims to implement a binary classification solution for the detection and classification of kidney tumors. Artificial neural network modeling effectively detects tasks and categorizes objects, image classification, and segmentation. The use of CNN in such a case helps to identify the feature map for each image engaged in the tanning process for the adopted CNN model. As represented in Figures 15 and 16, two categories are used to be trained for each phase. In the first phase, we classify the case as; Normal case, or Tumor case, while in the second phase, we classify the detected tumor as Benign tumor or Malignant tumor.

The attribute of our interest in the first phase is the “situation,” which is shown in Table 4. It comprises different values that are merged to balance the number of labels in the first case of detection of the tumor. We have merged the situation for the normal cae “healthy” and normal case with the cyst, as “Normal” of the tumor (Normal = 0) label and the situation of tumors as “tumor” (Tumor = 1) label. Finally, the attribute comprised new binary labels (0 and 1).  Table 10 shows the new labels.

The attribute of our interest in the second phase is the “tumor type,” which is shown in Table 5, we present the benign tumor as (benign = 0) label and the malignant of tumors as (malignant = 1) label. Finally, the attribute became composed of new binary labels (0 and 1).  Table 11 shows the new labels.

### 4.1. Data Preprocessing and Augmentation

#### 4.1.1. Preprocesses

Each patient had a file containing a video of a CT scan, where the number of pictures in the videos for patients varied, from 200 *±* 900 images. As an initial step, the video was divided manually into frames. In addition, clinical imaging data were stored and transmitted in the DICOM format. We converted images from the complex DICOM format to JPEG format, much smaller and easier to use [41]. After converting the image format, 70 images were chosen for each patient that showed the kidneys from different dimensions. Besides, for metadata, we have used the OpenRefine tool and tableau to make some preprocesses steps, having a cleaned text dataset to make visualization for data. See Figure 14.

#### 4.1.2. Image Normalization

We normalize the images by resizing the layers from 3 to 1 channel (converting RGB image into a grayscale). We also normalize the image size; the CT window level and breadth were set to emphasize the renal area while suppressing information from other organs and tissue.

This step of normalization is Figure 17 by reshaping the images to the preferred size of 224 × 224; this allows the network to acquire adequate renal context information from CT volumes. Reducing the image size is important because sometimes the image contains a lot of information; we can remove this kind of redundant important information.

#### 4.1.3. Feature Extraction

We have used OpenCV for image scans, which is a large open-source toolkit that supports *Python* language. It can detect objects from images and videos. In addition, OpenCVhas an algorithm named Canny, which provides the ability to extract image edge features [42]; see Figure 18.

Figure 18 shows an example of output for the Canny edge detector on one of the dataset images. We can notice that it provides a deep level of information, especially between the separations of the kidney. From this view, we can see that before training models, we have to use data augmentation to increase our dataset series of images per epoch in the training model, to enhance the model's generalization capability. In this way, the CNN will be able to distinguish this feature by its deep layers epoch by the epoch of learning; by this analysis, we discover that we need to use data augmentation.

#### 4.1.4. Image Augmentation

Preprocess improves the accuracy of the proposed methodology by normalizing and augmenting data. Image data augmentation is used to boost the model's learning capabilities and generalize its performance. Augmentation is a technique for artificially increasing a training dataset's size by producing updated images in the dataset. The data augmentation class can be specified once the data I/O interface has been initialized [43]. Data augmentation is a powerful technique to minimize model error rate (overfitting) by expanding training data. The used metrics in augmentation are

- Re-scale: it is used with the aim to scale the 255 values to the static range (224 × 224).
- Shear range: the image will be distorted along an axis, mostly to create or rectify the perception angles. We used 0.2 on the original image.
- Zoom range: the amount of zoom is 0.2 on the original image.
- Horizontal flip: we flipped the images horizontally.

Figure 19 shows an example of generating four new images based on the original CT. These valuable techniques are commonly used to create synthetic data, train large neural networks, and make our proposed models more robust to avoid overfitting when training the deep learning model. Also, when we face data scarcity, if the number of patients in the data set is minimal, it can be adjusted by rotation, reflection, etc. As a result, we get entirely new and manufactured images using different technologies.  Figure 20 shows an example of applying augmentation operations in Renal CT.

Image data augmentation is supported in the Keras deep learning library via the ImageDataGenerator class. Usually, image data augmentation is applied only to the training data set, not to the validation or test data set. In addition, it may be useful to try data augmentation methods separately to see if they lead to a measurable improvement in model performance, perhaps using a small sample data set and a model and a training run. Finally, following the process of augmenting the dataset, an augmented dataset was acquired. The data size of the tumor detection task before applying the augmentation method was 8400, and it was increased by four times, after the increase it became 33,600. Also, the data size of the tumor type classification task before applying the augmentation method was 4200 and it was increased by four times, after the increase it became 16,800. Thus, this data increases the performance of our models, especially when the available dataset is unbalanced. Also, augmentation reduces the training time, the model error rate, and the accuracy of classification tasks.

### 4.2. Building Models

This section describes the detection and classification models architecture used to predict four outputs; first, the normal case and the tumor case, then, the benign tumor and the malignant tumor. We have built four models; VGG16, ResNet50, and two modified CNN.

#### 4.2.1. VGG16 Detection Model

The network architecture consists of 16 layers deep: 13 convolutions 4 max-pooling and 3 fully connected layers. The convolutional input layer has a shape of 224 × 224 × 3; this layer determines the input dimensions and shape. Max-pooling minimizes the dimensionality of images by reducing the number of pixels from the previous convolutional layer. In addition, a fully connected ANN has an input layer that reflects the size of max-pooling output data and a hidden layer with the Relu activation function, also an output layer with a softmax output classifier that performs the prediction percentages for each class.  Figure 21 shows the network structure of the VGG16 architecture.

#### 4.2.2. ResNet50 Detection Model

The network architecture consists of 50 layers deep, 49 convolutions and one fully connected layer. The convolutional input layer also has a shape of 224 × 224 × 3, which is the maxpooling layer of images. The fully connected network, which has an input layer that reflects the size of the max-pooling output data and a hidden layer with the Relu activation function, also has an output layer with a Softmax output classifier that performs the prediction percentages for each class.  Figure 22 shows the network structure of the ResNet50 architecture.

#### 4.2.3. CNN-6 Detection Model

The proposed model for the detection of the tumor consists of 6 deep CNN layers with fully connected ANN. First is the batch normalization layer, which standardizes the inputs to a layer for each minibatch. By this, the model can reduce overfitting and enhance classification accuracy. Then, the convolution 2D input layer, represented as an input layer in 2D, creates a convolution kernel that works with layers input to produce a tensor of outputs. The Kernel is a convolution mask that can be used for blurring, sharpening, embossing, edge detection, and so on as a features extractor from the original image with the help of other layers. It is important to note that there is no difference between 1D, 2D, or 3D except in the number of dimensions.

Conv2D took several parameters that specified its working process. As an example, modelName.add (Conv2D (32, (3, 3), input shape = (224, 224, 3), activation = “Relu”)), which means that the Conv2D will learn a total of 32 filters after that the use of use max-pooling layer is to reduce the spatial dimensions of the output features data volume. This value is usually used as a value of power. The other parameter is the kernel size (3 × 3), where we define the kernel dimensions. The dimension must be a two-dimensional array of an odd number to specify the height and width of the 2D convolution frame applied to the original image to extract the features from it. While the activation = Relu (rectified linear activation function) defines the activation function that we want to apply on this input layer defined as *y* = max (0, *x*). It also might be softmax, which is more suitable for output activation in binary classification and low target classes such as 2 or 4. The softmax function is a function that turns a vector of *K* real values into a vector of *K* real values that sum to 1.

The input values can be positive, negative, zero, or greater than one, but the softmax transforms them into values between 0 and 1 to be interpreted as probabilities. If one of the inputs is small or negative, the softmax turns it into a small probability, and if the input is large, it turns it into a significant probability. Still, it will always remain between 0 and 1.

The input shape is the primary parameter for this layer where it defines the structure for the input image formulated as Image Width × Image Height × Image Channels in this example (224 × 224 × 3). Then is the Max-Pooling2D layer 2 × 2; this max-pooling is a type of operation that is typically added to CNN's following individual convolutional layers. When added to a model, max-pooling reduces the dimensionality of images by reducing the number of pixels in the output from the previous convolutional layer.

Then, the dropout layer randomly sets input units to a value with a rated frequency at each step during training time. Thus, it helps to reduce model overfitting. Then, a flattened layer flattens its input into a flatted output such as 2D into 1D of values (2 × 2) input becomes four as output. Then, the dense layer, which defines the hidden layer or the output layer, takes the number of neurons and the activation function. In the output layer, the number of neurons matches the number of training classes.  Figure 23 shows the network structure of the modified CNN architecture.

The proposed model for detecting the tumor consists of 6 deep CNN layers with fully connected ANN: first, the batch normalization layer, which standardizes the inputs to a layer for each minibatch and then the convolution 2D input layer. The Kernel is a convolution mask that can be used for blurring, sharpening, embossing, edge detection, and so on. Conv2D took several parameters that are specific to its working process. Max-pooling layer is to reduce the spatial dimensions of the output features data volume. Next, the dropout layer helps to reduce model overfitting. Then, the flattening layer flattens its input into a flatted result. Then, the dense layer defines the feedforward network. In the output layer, the number of neurons much matches the number of training classes.  Figure 23 shows the network structure of the modified CNN architecture.

#### 4.2.4. CNN-4 Classification Model

The proposed model for the classification of the tumor type consists of 4 deep CNN layers with fully connected ANN: first, the convolution 2D input layer; then, Max-Pooling2D layer 2 × 2; after that, the flattening layer; and then, the dense layer. In the output layer, the number of neurons matches the number of training classes.  Figure 24 shows the network structure of the CNN architecture.

## 5. Experimental and Results

This section presents the experiments of four different models, VGG16, ResNet50, and two modified CNN. The four models were run with often the same hyperparameters, though all had different network architectures. Results are shown in the following subsections.

### 5.1. Experiments Setup

The proposed models have been implemented on Colab using *Python* Programming language libraries: Tensorflow, Keras, SKlearn, Optimizer, and Backend. Additionally, we have used several *Python* packages like OpenCV2 for image processing and image augmentation. All experiments have been performed on a workstation with *Python* 3 Google Compute Engine backend (GPU), (0.80 GB/12.69 GB of RAM), and (38.73 GB/68.35 GB of Disk).  Table 12 shows the parameter setting for our experiment details.

The parameters were selected based on the experiments, which gave us the best results for the parameters mentioned in Table 12. They were described in detail as the following:

- Stepper epoch: it defines the number of learning steps that will be done in each epoch. We need a high number of training steps in each epoch since our data are large, and in our data augmentation, we declare it based on the batch size, so we have to make the steps larger than the batch size.
- Epochs: it is the number of times the dataset is being completed to the network, which can help in reusing the same dataset for training again. An epoch means training the neural network with all the training data for one cycle.
- Validation steps: same as steps per epoch but in this case, it defines the number of validation samples applied to the model in each epoch to reduce loss and increase the accuracy of classification.
- Loss: it is the value that is calculated after each iteration to define the error, which is calculated by the loss function.
- Optimizer: it helps reduce the output error of the loss function by changing the weights and bias values in the model and computes the adaptive learning rates for each parameter in the training phases. In our adopted CNN tools, we have used Adam optimizer. We experimented with Adam and other optimizers and found that the use of Adam is more accurate, as it also proves that Adam is the best in image classification problems.
- Activation function: it is a function used to choose whether the neuron should fire the data or not by obtaining the value received from the neuron and reevaluating it.
- Learning rate: it is a factor that is used along with the optimizer in changing the weights of the function, to end up with high accuracy.
- Batch size: it is the number of samples processed before the model is updated. It must meet the data sample but we reduce this number since our feature vector represents the image itself without a region of interest information so there is no need to take a high number of batches.
- Input neuron: it receives the image binary data as a feature vector. According to the image size 224 × 224, we found that 32 is the best number for our model training.
- Hidden neuron: it is trained on the input images to build the training model. We took the number of neurons in the input layer and multiply it by the number of image channels and increased the value to 128 to enhance the processing time.
- Output neuron: it defines the output classes that we have.

### 5.2. Adopted Experiment Dataset

For the detection task, the collected data were divided into 80% for the training set and 20% for the testing set. The training dataset was also divided into training and validation, which consisted of 5376 images for train and 1344 for validation. At the same time, the total number of images for testing is 1680. On the other hand, the training dataset used in the classification model for the kidney tumor type consists of 2688 images. Therefore, the total number of images for validation is 672. At the same time, the total number of images for testing is 840.

For the detection task, the collected data were randomly divided into 80% for the training set and 20% for the testing set. The training dataset was also divided into training and validation, which consisted of 5376 images for train and 1344 for validation. At the same time, the total number of images for testing is 1680.  Table 13 represents the values with the dataset splitting percentages.

The training dataset used in the classification model for the kidney tumor type consists of 2688 images. The total number of images for validation is 672. At the same time, the total number of images for testing is 840.  Table 14 represents the values with the dataset splitting percentages.

### 5.3. Evaluation Metrics

Based on the preprocessed dataset, we have used the confusion matrix [44] to evaluate our networks. We have used *F*-score metrics, which being calculated from the precision and recall of the test phase. More details about evaluation metrics are as follows:

- True Positive (TP): it represents the correctly predicted positive values, which means that the value of the actual class is yes, and the value of the predicted class is also yes.
- True Negative (TN): it represents the correctly predicted negative values, which means that the actual class's value is no, and the value of the predicted class is also no.
- False Positive (FP): it is when the actual class is no, and the predicted class is yes.
- False Negative (FN): it is when the actual class is yes but the predicted class is no.
- Accuracy: this is a performance measure, which is the number of correct predictions (Accuracy = TP + TN/TP + FP + FN + TN).
- Precision: it is the ratio of correctly predicted positive observations to the total predicted positive observations (Precision = TP/TP + FP).
- Recall (sensitivity): it is the ratio of correctly predicted positive observations to all observations in actual class (Recall = TP/TP + FN).
- F1 score: it is a measure that provides a single score that balances both the concerns of precision and recall in one number (F1 Score = 2 × (RecallxPrecision)/(Recall + Precision)).

### 5.4. VGG16 Detection Model Training and Testing

Training the VGG16 model on the data produced a loss value of 0.3506 and a test accuracy of 0.5938.  Figure 25 represents the loss and accuracy for both training and validation during the training process through each epoch. The values show how stable the model is.

The model was tested on 848 samples from the normal class and 832 samples from the tumor class. For normal cases, the model was able to classify 764 samples correctly, while it failed in 84 samples. However, for tumor cases, it classified 585 samples correctly while it failed in 247 samples.  Table 15 shows F-score diagnostic testing.

The training accuracy of ResNet50 reached 0.60, while the test accuracy reached 0.5938. Loss value implies how well or poorly a certain model behaves after each iteration of optimization. The value of the test loss in the VGG16 model is 0.3506, and the training time is 3 s 68 ms/step. From the previous results, we can conclude that the VGG16 model is weakly trained, and it behavior was poor in the testing process.

### 5.5. ResNet50 Detection Model Training and Testing

Training the ResNet50 model on the data produced a loss value of 0.0806 and a test accuracy of 0.9747.  Figure 26 represents the loss and accuracy for both training and validation during the training process through each epoch. The values show how stable the model is.

The model was tested on 848 samples from the normal class and 832 samples from the tumor class. For normal cases, the model was able to classify 806 samples correctly, while it failed in 42 samples. However, for tumor cases, it classified 813 samples correctly while it failed in 19 samples.  Table 16 shows *F*-score diagnostic testing.

The training accuracy of ResNet50 reached 0.96, while the test accuracy reached 0.9747. Loss value implies how well or poorly a certain model behaves after each iteration of optimization. The value of the test loss in the ResNet50 model is 0.0806, and the training time is 3 s 70 ms/step. From the previous results, we can conclude that the ResNet50 model is well-trained, and it behavior was good in the testing process.

### 5.6. CNN Model Detection Training and Testing

Applying the CNN model, the loss reached 0.1480, which is the distance between the actual values of the problem and the values predicted by the model. The test accuracy is 0.9531.  Figure 27 shows the loss and accuracy for both training and validation during the training process for each epoch.

The test was performed on 848 samples from the normal class and 832 samples from the tumor class. The model was able to classify 823 samples correctly while it failed in 25 samples. On the other hand, tumor classifies 801 samples correctly while it fails in 31 samples.  Table 17 shows *F*-score diagnostic testing.

The training accuracy, which is the accuracy of the CNN model, reached 0.97. The test accuracy reached 0.9531. Moreover, the loss value implies how well or poorly a certain model behaves after each optimization iteration. The value of the test loss in the CNN detection model is 0.1480. At the same time, the training time is 3 s 62 ms/step. From the previous results, we can conclude that the CNN model is well-trained, and it performed exemplary in the testing process.

### 5.7. CNN Model Classification Training and Testing

After performing a CNN model training based on the previous data mentioned above, we got a loss of 0.0643 and an accuracy of 0.9777. We also got the following graph representing the loss and accuracy for both training and validation during the training process through epochs. The values show how stable the model is in Figure 28.

The test was performed upon 531 samples from the malignant class and 234 samples from the benign class. For the malignant class, the model was able to classify 229 samples correctly while it failed in 5 samples. On the other hand, for benign, it correctly classifies 474 samples while it fails in 57 samples.  Table 18 shows *F*-score diagnostic testing.

The training accuracy for this model reached 0.9777. The test accuracy reached 0.92. At the same time, the training time is 1 s 64 ms/step.

Table 19 shows the accuracy, training loss, number of epochs, and training time, for all proposed deep learning models where three models were used for tumor detection and one model for tumor classification. Based on the models that we built, we can say that they are promising in diagnosing kidney tumors because of their high accuracy in diagnosis.

## 6. Comparison with Other Related Studies

In comparison with the previous works, the proposed methodology and the 2D-CNNs have achieved fruitful results by using CT scans for kidney patients. This is the first research for the detection and classification of kidney tumors based on the new data, which can help doctors and radiologists find the appropriate treatment plan for kidney tumor patients. According to the data in Table 20, which represents a comparison between our proposed work and the previous work, our research is considered the first research that utilized bigger data of CT scans. Moreover, it has outperformed the previous works in accuracy reaching a 97% score for tumor detection and a 92% score for tumor classification.

The results of previous studies proved the power of using deep learning approaches in renal tumor detection and classification tasks. Researchers in the other studies have operated practical methodologies for a fair comparison and achieved satisfactory results. One of the challenges that researchers faced was the availability of data. Usually, the data on medical images are few in terms of numbers, which leads to high risks of overtraining and subsequently reduced performance. Some solutions that can help mitigate this problem are using smaller models and augmenting the data. Also, there is more than one study on the same dataset, which affects the limitations of the studies. Because of the challenges of collecting and building data, it takes time and effort, especially pulling the data. In addition, it must be ensured that the data are properly structured in continuous cooperation with specialists. Although obtaining new data is difficult, there is a need for a new expanding dataset to perform a complete diagnosis that covers the limitations of the diagnosis to cover all aspects of diagnosis, not only tumor detection and classification of tumor type but also for classification of tumor subtypes, stage, and segmentation in one operation.

## 7. Discussion and Conclusion

This paper uses four methods, VGG16, ResNet50, and two different modified 2D-CNN models, to study the patient's situation with kidney tumor injury and define the kidney tumor type. Based on renal CT scans, the features extracted helped recognize the image class (Normal/Tumor and Benign/Malignant) by training and testing methods. For our novel dataset, the results proved the effectiveness of our proposed 2D-CNN models, where the accuracy for the detection models VGG16, ResNet50, and 2D-CNN reached 60%, 96%, and 97%, respectively. On the other hand, the classification 2D-CNN model got 92%.

For revealing the specific characteristics of a kidney tumor, the data of patients need to be collected. After all, the process of labeling, building data, and converting the image format takes time. In addition, the images are drawn manually for each patient and need to cooperate with radiologists to validate the data. Several of the previous studies did not take more than one image of the patient. As a result, there are limitations in the diagnosis and studies; ideally, the data set should be more extensive. Thus, the precise composition of our data set is impressive since it does not contain missing data and carries valuable information from the metadata. Besides, the images cover multiple aspects of diagnosis. There are 70 images for each patient in which kidney problems can be predicted, including tumors and stones, cysts, and other tumors in the nearby organs.

Some challenges were encountered in this study, summarized in several points; a process of manually data collection, segmenting video and converting the image from DICOM to JPEG, image selection, text data building, data labeling, and missing data, where we encountered technical problems and re-collected data for some patients, overfitting problems, and the need for high-performance servers.

The main contributions of this paper can be summarized as follows: originating new datasets from a Jordanian hospital consisting of text data of clinical reports and sequences images of CT scans, a case study, and statistical analysis of kidney tumor cases in one of the most important hospitals in northern Jordan, exploring the performance of the modified 2D-CNN models for the tumor detection and classification task, enhancing the diagnosis of patient conditions with high accuracy, reducing the doctor's and radiologist's workload, and providing them with a tool that can automatically assess the condition of the kidneys, support a better understanding of the evaluation results, and predict the presence of tumors in any patient. Besides, the results of the models can reduce the risk of misdiagnosis. Furthermore, increasing the quality of healthcare service and early detection can change the disease's track and preserve the patient's life.

Our future work includes further optimizing the detection performance and accurate extraction of renal tumors from CT scans and additionally making classification tasks for the tumor subtypes that we have identified and other multiple diagnostic studies such as classifying tumor stage and segmenting the tumor in both kidneys. We look forward to having a full diagnosis of this new data toward having a robust standard for intelligent diagnosis of kidney tumors.

## Figures and Tables

**Figure 1:** Sample renal CT taken from the dataset.

**Figure 2:** Architecture of a traditional CNN.

**Figure 3:** VGG16 architecture.

**Figure 4:** ResNet50 architecture.

**Figure 5:** Sample CT scans taken from the dataset.

**Figure 6:** An analysis of gender and situation for all cases in the dataset.

**Figure 7:** An analysis of age for healthy and tumor patients.

**Figure 8:** Numbers of healthy and tumor patients who took a contrast.

**Figure 9:** An analysis of the classification of kidney tumor type.

**Figure 10:** An analysis of the classification of kidney tumor subtype.

**Figure 11:** An analysis of gender and classification of kidney tumors type.

**Figure 12:** Statistical analysis for tumor segmentation in both kidneys.

**Figure 13:** An analysis of tumor type and stage.

**Figure 14:** Methodology diagram.

**Figure 15:** Detection labels.

**Figure 16:** Classification labels.

**Figure 17:** An overview of the normalization step.

**Figure 18:** Original input CT images and edge detector output images.

**Figure 19:** The augmentation techniques used.

**Figure 20:** An example of applying augmentation operations.

**Figure 21:** Schematic representation of the VGG16 architecture of detection kidney tumor.

**Figure 22:** Schematic representation of the ResNet50 architecture of detection kidney tumor.

**Figure 23:** Schematic representation of the CNN architecture of detection kidney tumor.

**Figure 24:** Schematic representation of the CNN architecture of classification kidney tumor type.

**Figure 25:** Evaluation results for the VGG16 detection model.

**Figure 26:** Evaluation results for the ResNet50 detection model.

**Figure 27:** Evaluation results for the CNN detection model.

**Figure 28:** Evaluation results for the CNN classification model for tumor type.

**Table 1:** Current public CT datasets for kidney tumors.

Ref.	Dataset	Year	Type	Size	^#^Patient
[30]	G037-RCP: London	2017	CT	5,339	5,339
[31]	C4KC-KiTs19	2019	CT	210	210
[32]	TCGA-KICH	2020	CT	439	267
[33]	TCGA-KICH	2020	CT	15	15
[34]	TCGA-KIRP	2020	CT	47	33
[35]	CPTAC-CCRCC	2020	CT	670	63
[36]	KAUH: Jordan	2021	CT	8,400	120

**Table 2:** Statistical analysis of all patients' situations.

Gender	Normal “healthy”	Normal with cyst	Tumor
Male	15	12	38
Female	17	16	22
Total	**32**	**28**	**60**

**Table 3:** Dataset attributes' description.

^#^	Attribute	Description
1	Patient ID	ID
2	Patient num	Count
3	Age	Age
4	Gender	Sex
5	Test area	(Chest/abdomen/pelvis)
6	Date	Year
7	Taking contrast	Contrast material
8	Clinical data	Historical data
9	Symptoms	Symptoms before test
10	Diagnosing test	Full diagnosing
11	Diagnosing right kidney	Diagnosing RK
12	Injury range right kidney	Injury range in details
13	Segmentation injury in right kidney	Location injury in RK
14	Diagnosing left kidney	Diagnosing LK
15	Injury range left kidney	Injury range in details
16	Segmentation injury in left kidney	Location injury in LK
17	Stage	Out of IV
18	Situation	Kidney status
19	Tumor type	If malignant or benign
20	Tumor class	Tumor subtype

**Table 4:** Situation labels description.

Label	Description
Normal case “healthy”	The kidneys are healthy
Normal case with cyst	Other problems than tumor
Tumor	Kidney tumor injury

**Table 5:** Tumor type labels description.

Label	Description
Benign	Non-cancerous tumor
Malignant	Cancerous tumor

**Table 6:** Contrast label description.

Label	Description
Yes	Given contrast material before the test
No	Not given contrast material before the test

**Table 7:** Tumor classification labels description.

Label	Description
Adenoma	Benign
Angiolipoma	Growth made of fat and blood vessels
Lipomas	Fatty tumor
RCC	Renal cell carcinoma
Secondary	Metastasis from other organs

**Table 8:** Stage labels description.

Label	Description
I	7 cm or less, only affects the kidney, has not spread
II	Greater than 7 cm, only affect the kidney, has not spread
III	Grown to blood vessels, may spread in around
IV	Tumors spread into the adrenal gland or to other organs

**Table 9:** Segmentation of the injury in the right and left kidney labels description.

Label	Description
Upper	Tumor in the upper part of the kidney
Middle	Tumor in the middle part of the kidney
Lower	Tumor in the lower part of the kidney
Healthy	There is no tumor
Undefined	Partial, nephrectomy, blurred kidney, undiagnosed

**Table 10:** Situation attribute labels merged description.

Label	Description
0	Normal
1	Tumor

**Table 11:** Tumor type labels merged description.

Label	Description
0	Benign
1	Malignant

**Table 12:** Models parameter.

Parameter	Value
Step_Per_Epoch	Training images/batch size
Epochs	VGG16: 44, ResNet50: 25, CNN's: 50
Validation steps	Validation images/batch size
Loss	Binary cross entropy
Optimizer	Adam, SGD
Activation function	ReLu, Sigmoid, Softmax
Learning rate	0.001
Batch size	32
Input neuron	32 shape of 224 × 224
Hidden neuron	128
Output neuron	2

**Table 13:** First phase values with the dataset splitting percentages of totally 8400 images.

Dataset	Number	Splitting factor
Training	5376	Training 80%
Validation	1344	—
Testing	1680	Testing 20%

**Table 14:** Second phase values with the dataset splitting percentage of totally 4200 images.

Dataset	Number	Splitting factor
Training	2688	Training 80%
Validation	672	—
Testing	840	Testing 20%

**Table 15:** Accuracy results achieved by the VGG16 model.

ResNet50	Precision	Recall	F1	Accuracy
Normal	0.57	0.90	0.7	**0.60**
Tumor	0.75	0.30	0.42	

**Table 16:** Accuracy results achieved by ResNet50 model.

ResNet50	Precision	Recall	F1	Accuracy
Normal	0.98	0.95	0.96	**0.96**
Tumor	0.95	0.98	0.96	

**Table 17:** Accuracy results achieved by CNN detection model.

CNN	Precision	Recall	F1	Accuracy
Normal	0.96	0.97	0.97	**0.97**
Tumor	0.97	0.96	0.97	

**Table 18:** Accuracy results achieved by CNN classification model.

CNN	Precision	Recall	F1	Accuracy
Benign	0.99	0.89	0.94	**0.92**
Malignant	0.80	0.98	0.88	

**Table 19:** An overview of training and testing of accuracy, loss, epochs, and time for all models.

Model	Testing	Training	Loss	Epoch	Time
VGG16	0.593	0.60	0.3506	44	3 s 68 ms/step
ResNet50	0.974	0.96	0.0806	25	3 s 70 ms/step
CNN-6	0.953	0.97	0.1480	50	3 s 62 ms/step
CNN-4	0.977	0.92	0.0643	50	1 s 64 ms/step

**Table 20:** Overview of the related studies about kidney tumor detection and classification based on CT scans.

Ref.	Year	Source	Size	Methods	Result
[23]	2014	India		SOM, ANN	85%
[24]	2014	US	167	HOG, MMD, SURF	95%
[25]	2015	India	28	ASNN, KNN	
[27]	2020	US	315	CNN	83%
[26]	2019	China	192	ROC, InceptionV3	97%
[28]	2020	Canada	177	XGBoost	70%, 77%
[29]	2020	US	735	AdaBoost, RF	68–75%
[36]	**2021**	Jordan	**8400**	2D-CNN	**92%, 97%**

## Data Availability

Data are available from the authors upon reasonable request.
